The article "Characteristics of the Dynamic Electrocardiogram in the Elderly with Nonvalvular Atrial Fibrillation Combined with Long R-R Intervals" was retracted in 2023. Reasons: unreliable results or conclusions; lack of ethics approval or compliance; concerns about the data; concerns about the peer review.

# Characteristics of the Dynamic Electrocardiogram in the Elderly with Nonvalvular Atrial Fibrillation Combined with Long R-R Intervals

**DOI:** 10.1155/2021/4485618

**Published:** 2021-11-10

**Authors:** Hongyuan Xu, Jinyi Li, Guoqiang Zhong, Lin Li, Chuang Huang, Peng Guo, Yizhao Chen, Tao He

**Affiliations:** ^1^Cardiology Department, The Eighth Affiliated Hospital of Guangxi Medical University, Guigang, Guangxi 537100, China; ^2^Cardiology Department, The First Affiliated Hospital of Guangxi Medical University, Nanning, Guangxi 530021, China; ^3^Cardiology Department, Affiliated Hospital of Guilin Medical University, Guilin, Guangxi 541001, China; ^4^ECG Diagnosis Department, The First Affiliated Hospital of Guangxi Medical University, Nanning, Guangxi 530021, China

## Abstract

**Objective:**

To investigate the characteristics of dynamic electrocardiogram and their clinical implications in elderly patients with nonvalvular atrial fibrillation combined with long R-R intervals.

**Methods:**

Elderly patients diagnosed with nonvalvular atrial fibrillation who were admitted as an inpatient or attended the outpatient department from January 2015 to January 2020 were selected. Patients were divided into two groups based on the presence of a long R-R interval. The characteristics and therapeutic significance of dynamic electrocardiogram between the two groups were compared.

**Results:**

A total of 532 patients were included in our analyses. Of these, 399 patients were in the long R-R interval group and 133 in the nonlong R-R interval group. In 399 patients, there were 48,840 long R-R intervals manifested within 24 hours. The average, slowest, and fastest ventricular rates during sleep time were higher than those in nonsleep time, while the number of long R-R intervals in sleep time was significantly smaller than that in nonsleep time (*P* < 0.05). Clinical parameters including dizziness/syncope, cerebral infarction, ST-segment changes, platelet count, average hematocrit, prothrombin time (PT), left ventricular systolic function, end-diastolic diameter, pulmonary artery pressure, and left ventricular ejection fraction were comparable between the groups (*P* > 0.05). When compared with the nonlong R-R interval group, the level of C-reactive protein was slightly lower in the long R-R interval group (*P* < 0.05). In addition, the long R-R interval group had a higher incidence of atrial premature beats but a lower incidence of ventricular premature beats. Furthermore, the probability of long R-R interval combined with paroxysmal atrial tachycardia, transient ventricular arrest, second-degree atrioventricular block, and complete or incomplete right bundle branch block was higher than that of nonlong R-R interval (*P* < 0.05). In patients with long R-R interval >3 s, the risk of having second-degree atrioventricular block and complete or incomplete right bundle branch block was significantly lower, while the risk of having transient ventricular arrest was higher when compared to patients with long R-R intervals of 2-3 s (*P* < 0.05*P*).

**Conclusions:**

Long R-R interval is a common electrocardiographic phenomenon among the elderly with nonvalvular atrial fibrillation. The long R-R interval mostly occurs in nonsleeping time. The average ventricular rate, slowest ventricular rate, and fastest ventricular rate of sleep time are higher than nonsleeping time. Analysis of the characteristics of the dynamic electrocardiogram of these patients may shed light on the mechanisms for long R-R intervals, including the likelihood of concealed conduction and physiological interference in the atrioventricular node, overspeed inhibition, increased vagus nerve tension, or pathological atrioventricular block.

## 1. Introduction

As one of the most common cardiovascular diseases, atrial fibrillation is widely observed among the elderly with the incidence of 2–4% and 8% in those aged over 60 and 80 years, respectively [1, 2]. Given the aging population, the incidence of atrial fibrillation continues to increase drastically in recent decades. Nonvalvular atrial fibrillation represents the most common type that accounts for 87.0% of all cases of atrial fibrillation. Patients with nonvalvular atrial fibrillation are highly susceptible to thromboembolism. Also, the continuous elevated atrial pressure promotes sympathetic activity, resulting in a vicious circle of atrial fibrillation with heart failure and consequently a high fatality rate among patients with nonvalvular atrial fibrillation [2, 3].

Long R-R interval, defined as > 1.5 s, is commonly observed in the dynamic electrocardiogram of patients with atrial fibrillation. Atrial fibrillation is more likely to occur with a significantly prolonged R-R interval when compared with sinus rhythm, for which a standard of >2.0 s is widely applied in clinical practice [4, 5]. Therefore, the dynamic electrocardiogram is the main diagnostic method for long R-R intervals; the frequency, temporal distribution of the occurrence, and heart rate variability of long R-R intervals are shown by continuous monitoring over 24 hours. To date, guidelines on the optimal clinical management of this cardiac electrical phenomenon are lacking, with the restoration of sinus rhythm being the best achievable outcome. Removal of triggers and factors causing persistent AF is key for successful treatment. Therefore, in this study, the characteristics of dynamic electrocardiogram and their clinical implications in elderly patients with nonvalvular atrial fibrillation combined with long R-R intervals were analyzed ad compared with those without long R-R intervals.

## 2. Methodology

### 2.1. Patients

Elderly patients diagnosed with nonvalvular atrial fibrillation who were admitted as an inpatient or attended the outpatient department from January 2015 to January 2020 were selected. Patients were divided into two groups based on the presence of a long R-R interval.

The inclusion criteria of this study were as follows: (1) patient with a confirmed diagnosis of nonvalvular atrial fibrillation based on comprehensive examinations including clinical manifestation and dynamic electrocardiogram, and all patients had clinical symptoms such as dizziness, shortness of breath, and palpitations; (2) an R-R interval exceeded 2.0 s on continuous monitoring by dynamic electrocardiogram; (3) not consuming any medications that might affect the characteristics of electrocardiogram within 4 weeks prior to the inclusion in this study.

Patients were excluded if (1) diagnosed with ischemic cardiomyopathy, valvular rheumatic heart disease, congenital heart disease, or other severe organic heart diseases; (2) previously underwent valve replacement procedure or had acute decompensated heart failure; (3) presence of abnormal liver and kidney functions, bleeding disorders, systemic infectious diseases, chronic wasting diseases, or malignancies; (4) pregnancy and breast-feeding special population; (5) withdraw or terminate the study halfway; (6) history of mental illness.

This study was approved by the Medical Ethics Committee of the First Affiliated Hospital of Guangxi Medical University.

### 2.2. Investigations

Basic demographics of all patients in addition to clinical parameters such as biochemical results, coagulation profiles, and routine blood indices were collected.

Dynamic electrocardiogram characteristics were recorded using the ECGLAB dynamic electrocardiogram analysis system (Beijing MEIGAOYI Software Technology Co., Ltd.). The data were analyzed electronically and manually inspected to remove false differences. A detailed 24-hour activity log and the symptoms of patients were recorded. Dynamic electrocardiograms such as occurrence frequency and time of long R-R interval, fastest ventricular rate, slowest ventricular rate, and average ventricular rate of all patients were analyzed. For comparative analyses, patients were divided into the long R-R interval group and nonlung R-R interval group. Patients with long R-R intervals (≥2 s) were further divided into groups with R-R intervals of > 3 s or 2-3 s. The clinical manifestations and characteristics of the dynamic electrocardiogram between the groups were compared.

### 2.3. Statistical Analysis

SPSS 20.0 was used for statistical analysis. Continuous and categorical variables were presented as ($\bar{x}$ ± *s*) and compared with the *t*-test, while categorical variables were presented as rate (%) and compared with the *χ*^2^ test. A *P* value of <0.05 was considered statistically significant.

## 3. Results

A total of 532 patients were included in our analyses. Of these, 399 patients were in the long R-R interval group and 133 in the nonlong R-R interval group. The basic demographics of patients between the 2 groups were comparable (*P* > 0.05) (Table 1).

### 3.1. Characteristics of Dynamic Electrocardiogram

Of 399 patients with long R-R intervals, 254 and 154 had long R-R intervals of 2-3 s and >3 s, respectively. A total of 48,840 long R-R intervals were identified in the dynamic electrocardiogram of 399 patients within 24 hours. The majority of long R-R intervals occurred during the nonsleep time (75.32%), whereby midnight 6 am had significantly the lowest incidence of R-R interval when compared with those during 7 am–noon, 13 pm–18 pm, and 19 pm–23 pm (Figures 1 and 2, Supplementary Tables 1 and 2). Furthermore, the difference in the average, slowest, and fastest ventricular rates of patients between sleep time (9:30 pm–6:30 am) and nonsleep time (6:31 am–9:29 pm) was significantly different (*P* < 0.05) (Table 2).

### 3.2. Characteristics of the Electrocardiogram of Patients with Long R-R Interval ≥2 s

Of 399 patients with long R-R interval, 124 (31.08%) and 15 (3.76%) had ≥100 and ≥1000 long R-R intervals, respectively, in 24 h, and 45 (36.29%) were found to have a second-degree atrioventricular block. The maximum number of long R-R intervals was 5520 in 24 h.

### 3.3. Clinical Manifestation and Characteristics of Dynamic Electrocardiograms between the Groups

No significant difference was observed in the incidence of dizziness/syncope and the combination with cerebral infarction, ST-segment alteration, and ventricular premature beats between the groups (*P* > 0.05) (Table 3). However, the long R-R interval group had a significantly higher incidence of atrial premature beats (*P* < 0.05).

### 3.4. Clinical Parameters and Combination with Other Arrhythmias

Parameters including platelet count, mean hematocrit, prothrombin time (PT), left ventricular internal diameter at end-systole and end-diastole, pulmonary artery pressure, and left ventricular ejection fraction of both groups were comparable (*P* > 0.05) (Table 4). The level of C-reactive protein in the long R-R interval group was significantly lower than that in the nonlong R-R interval group (*P* < 0.05).

When comparing other arrhythmias between the groups, the probability is that the long R-R interval group had significantly higher incidences of paroxysmal atrial tachycardia, paroxysmal atrial flutter, transient ventricular arrest, second-degree atrioventricular block, complete or incomplete right bundle branch block (*P* < 0.05) (Table 5).

### 3.5. Characteristics of Dynamic Electrocardiograms of Patients with Long R-R Intervals (2-3 s vs. >3 s)

Of 399 patients with long R-R interval, 154 had the R-R interval of >3 s, while 245 had intervals of 2-3 s (Table 6). The proportions of patients with second-degree atrioventricular block, paroxysmal atrial tachycardia, transient ventricular arrest, and complete or incomplete right bundle branch block were significantly lower in patients with long R-R intervals of >3 s than those with intervals of 2-3 s (*P* < 0.05).

## 4. Discussion

Dynamic electrocardiogram can effectively detect atrial fibrillation with long R-R interval. The possible reason is that atrial fibrillation usually leads to atrial anatomical and electrophysiological remodeling, with the frequency of the f-wave at 350–600/min propagating to the ventricle only at a 2 : 1–5 : 1 ratio. The majority of nonvalvular atrial fibrillation have varying degrees of concealed conduction at the atrioventricular junction or with physiological interfering factors that render the atrial fibrillation wave unable to propagate to the ventricle, resulting in the emergence of a long R-R interval, and dynamic electrocardiogram can timely capture the changes of the atrium with the help of a computer [6]. The characteristics of dynamic electrocardiograms in this study suggested the phenomenon of mostly physiological rather than of true atrioventricular block. Also, the duration of long R-R intervals does not truly reflect atrioventricular conduction but may be the result of an f-wave concealed conduction (Supplementary Figures 1 and 2). Patients with long R-R intervals may have aggravated coronary heart disease and heart failure, in addition to increased risks of various other cardiovascular diseases that will impact clinical treatment. Therefore, continuous 24-hour dynamic electrocardiogram recording of patients with AF helps to identify abnormalities that are otherwise difficult to detect by routine electrocardiogram [7, 8].

In this study, a total of 48,840 long R-R intervals were identified in the dynamic electrocardiogram of 399 patients within 24 hours, and the majority (*n* = 36787, 75.3%) of long R-R intervals were observed during the nonsleep time, with the lowest number of R-R intervals observed during midnight 6 am. The average, slowest, and fastest ventricular rates in sleep time were higher than those in nonsleep time. Also, arrhythmias such as conduction block, paroxysmal atrial tachycardia, and ventricular tachycardia were only observed during sleep time in most patients. All these findings were consistent with previous studies [9], suggesting a significant change in the heart rate of patients during sleep time. Considering that the cardiac autonomic nervous system may have the same regulatory effect on the sinus and atrioventricular nodes, the ventricular rhythm in patients with atrial fibrillation also conforms to the circadian variation that is characteristic of cardiac homeostasis. Long R-R interval is correlated with sleep. The mechanism may be that the autonomic nerve regulates the heart, and the vagal nerve tension increases; when the human body is in sleep, the vagal tone is increased, which leads to decreased concealed conduction and refractory periods in the atrioventricular junction. This then drives the propagation of the f-wave to the ventricle, thereby reducing the atrioventricular nodal hidden conduction, further increasing the rate of atrioventricular impulse transmission down to the ventricle and leading to higher fastest and slowest ventricular rates compared with the nonsleeping states [10]. Additionally, we observed a paroxysmal increase in the long R-R interval when the patients were not in sleep, while some patients were found to have long R-R intervals both in sleep and nonsleep periods (Supplementary Figures 3 and 4). Therefore, the characteristics of the dynamic electrocardiogram we observed might be attributed to the coexistence of multiple mechanisms such as concealed conduction, physiological disturbance, and atrioventricular block. Prolonged atrial fibrillation induces anatomic and electrical remodeling of the atrial myocardium, leading to exacerbated persistent left atrial overload from left atrial internal diameter enlargement and consequently promoting the progression of paroxysmal to persistent atrial fibrillation despite the function of the sinus and atrioventricular node [11].

When comparing the long R-R interval group with the nonlong R-R interval group, our analyses did not reveal any significant difference in the incidence of some of the clinical parameters including dizziness/syncope, concurrent cerebral infarction, ST-segment changes, left ventricular internal diameter at end-systole and end-diastole, pulmonary artery pressure, and left ventricular ejection fraction, indicating that the occurrence of most long R-R intervals does not lead to significant hemodynamic changes or significantly affect the left ventricular structure or function. However, the level of C-reactive protein in the long R-R interval group appeared moderately lower than that in the nonlong R-R interval group (*P* < 0.05), suggesting some involvement of inflammatory response. Meanwhile, a higher incidence of atrial premature beats and a lower incidence of ventricular premature beats were observed in the long R-R interval group. In addition, the long R-R interval group had a significantly higher risk of other arrhythmias including paroxysmal atrial tachycardia, transient ventricular arrest, second-degree atrioventricular block, and complete or incomplete right bundle branch block than that of the nonlong R-R interval group, likely attributed to atrial fibrillation causing anatomic and electrical remodeling of the atrial myocardium as well as damage to the sinus node and atrioventricular node, which have relatively little effects on the ventricles. Further analyses have demonstrated that patients with long R-R interval >3 s had a significantly lower risk of having second-degree atrioventricular block and complete or incomplete right bundle branch block than those with long R-R interval of 2-3 s. Additionally, a longer R-R interval was associated with a greater risk of transient ventricular arrest and a decrease in second-degree AV block, which was mostly observed when atrial fibrillation returned to sinus rhythm, possibly as a result of “overdrive suppression” [12]. Paroxysmal atrial fibrillation and flutter are key indicators in evaluating the recovery of automaticity following overdrive suppression of the sinus node by a long R-R interval, and a long R-R interval of up to 3 s can be used to diagnose sick sinoatrial syndrome [13]. First, if the atrial fibrillation stops abruptly, the temporarily suppressed sinus node may lead to the appearance of a long R-R interval. Second, coronary ischemia results in amyloid changes in the sinus node or surrounding tissue, leading to fibrosis and degenerative changes in the sinus node, which makes the sinus node incompetent, and consequently the manifestation of a long R-R interval or sinus arrest. When “double nodes” lesions appear, ventricular escape or arrest is more likely to occur (Supplementary Figures 5–7). We also observed that in patients with long R-R intervals greater than 2 s, such intervals did not occur every day and their frequency also differed greatly. Meanwhile, the reverting of the long R-R interval resulting from each episode of atrial fibrillation to sinus rhythm varies, and even the first QRS front before reverting to sinus rhythm may be a sinus P wave or a junctional escape. All these shall be taken into consideration in the diagnosis of atrial fibrillation combined with second-degree atrioventricular block or deciding on the implantation of a permanent pacemaker (Supplementary Figures 8–10).

In summary, nonvalvular atrial fibrillation combined with long R-R interval is a common electrocardiographic phenomenon among the elderly. In the clinical management of such patients, the aims are to reverse the atrial fibrillation and maintain a sinus rhythm, control the ventricular rate, and prevent thrombosis. Sinus and atrioventricular node lesions will need to be considered during treatment. Analysis of the characteristics of dynamic electrocardiogram reveals several possible underlying mechanisms of long R-R interval: concealed conduction; increased vagal tone; anatomical and electrical remodeling of the heart due to atrial fibrillation, which affects the function of the sinus and atrioventricular node, resulting in sick sinus syndrome and atrioventricular block; atrioventricular junctional extrasystoles: inconsistencies in the layered conduction refractory period of atrioventricular junctions are important factors in generating irregular atrioventricular conduction ratios and long R-R intervals; “overdrive suppression:” the automaticity of the autonomous pacemaker sites is inhibited when the persistent fast-frequency stimulus enters the site of the autonomous pacing that is relatively slow in frequency, and its recovery cycle is significantly longer than the original cycle when the stimulus is terminated abruptly. Therefore, comprehensive analysis of multiple dynamic electrocardiograms helps to uncover the underlying mechanism, which allows the targeted management strategy to achieve an optimal clinical outcome in elderly patients with nonvalvular atrial fibrillation. To detect elderly nonvalvular atrial fibrillation with long R-R interval through dynamic electrocardiogram, it is necessary to pay attention to the time and frequency of long R-R interval and combine it with the patient's medical history, so as to provide an effective reference for clinical diagnosis and treatment and prognosis judgment. Clinicians should take active and effective measures to treat sleep-related and nonsleep-related people with different treatment plans to keep the ventricular rate within the normal range and further improve the quality of life of patients with cardiovascular diseases.

## Figures and Tables

**Figure 1:** The plot of frequency versus time period of long R-R interval in patients with nonvalvular atrial fibrillation.

**Figure 2:** Time period profiles of long R-R intervals in patients with nonvalvular atrial fibrillation.

**Table 1:** Basic demographics of patients in the long R-R interval group and nonlong R-R interval group.

Groups	Male/female	Age (mean, years)	History of smoking/alcohol consumption	Hypertension/diabetes/coronary heart disease	Duration of atrial fibrillation (mean, months)
Long R-R interval (*n* = 399)	276/123	73.52 ± 5.69	384/384	165/108/126	14.86 ± 5.68
Nonlong R-R interval (*n* = 133)	84/49	74.01 ± 5.70	128/126	65/48/20	15.01 ± 5.70
*χ* ^2^/*t*	1.386	0.860	0.069	2.002	0.264
*P*	0.239	0.390	0.792	0.157	0.792

**Table 2:** Characteristics of dynamic electrocardiograms of patients during sleep time and nonsleep time.

Groups	Number of long R-R intervals (*n* = 48,840)	Average ventricular rate (times/min)	Slowest ventricular rate (times/min)	Fastest ventricular rate (times/min)
Sleep time	12053 (24.68%)	82.56 ± 6.89	41.46 ± 6.47	155.52 ± 12.26
Nonsleep time	36787 (75.32%)	70.24 ± 8.51	35.51 ± 5.89	131.48 ± 10.87
*χ* ^2^/*t*	250.50.012	22.475	4.809	29.307
*P*	<0.001	<0.001	<0.001	<0.001

**Table 3:** Clinical manifestation and characteristics of dynamic electrocardiograms between the groups (*n* (%)).

Factor (*n* = 532)	Long R-R interval group (*n* = 399)	Nonlong R-R interval group (*n* = 133)	*χ* ^2^	*P*
Dizziness/syncope (*n* = 489)	372 (93.23%)	117 (87.97%)	3.045	0.081
Combination with cerebral infarction (*n* = 124)	94 (23.56%)	30 (22.56%)	0.014	0.906
ST-segment alteration (*n* = 348)	268 (67.17%)	80 (60.15%)	1.872	0.171
Combination with ventricular premature beats (*n* = 452)	335 (83.86%)	117 (87.97%)	0.961	0.327
Combination with atrial premature beats (*n* = 112)	96 (24.06%)	16 (12.03%)	7.977	0.005

**Table 4:** Clinical parameters of the long R-R interval group and nonlong R-R interval group.

Experimental parameters	Long R-R interval group (*n* = 399)	Nonlong R-R interval group (*n* = 133)	*t*	*P*
C-reactive protein (mg/L)	6.65 ± 1.27	9.38 ± 1.48	20.572	<0.001
Platelet count (10^9^/L)	195.45 ± 58.87	199.56 ± 61.24	0.690	0.490
Mean hematocrit (Fl)	90.12 ± 8.47	88.98 ± 10.14	1.277	0.202
Brain natriuretic peptide (pg/ml)	788.89 ± 124.56	805.56 ± 128.84	1.325	0.186
PT (S)	11.89 ± 2.49	12.01 ± 2.51	0.480	0.631
Left ventricular internal diameter at end-systole (mm)	33.10 ± 5.48	32.92 ± 5.51	0.328	0.743
Left ventricular internal diameter at end-diastole (mm)	50.35 ± 5.48	49.85 ± 5.51	0.910	0.363
Pulmonary arterial pressure (mmHg)	31.56 ± 12.14	30.05 ± 11.98	1.246	0.213
Left ventricular ejection fraction (%)	60.89 ± 10.24	61.23 ± 11.51	0.321	0.748

**Table 5:** Other arrhythmias of the two groups (*n* (%)).

Parameters (*n* = 532)	Long R-R interval group (*n* = 399)	Nonlong R-R interval group (*n* = 133)	*χ* ^2^	*P*
Second-degree atrioventricular block	45 (11.28%)	2 (1.50%)	10.650	0.001
Paroxysmal atrial tachycardia	35 (8.77%)	4 (3.01%)	4.067	0.044
Paroxysmal atrial flutter	68 (17.04%)	10 (7.52%)	6.490	0.011
Junctional escape beats	24 (6.02%)	9 (6.77%)	0.011	0.917
Ventricular escape beats	15 (3.76%)	5 (3.76%)	0.069	0.792
Linking phenomenon	8 (2.01%)	2 (1.50%)	0.136	0.712
Transient ventricular arrest	15 (3.76%)	0 (0.00%)	3.865	0.049
Accelerated ventricular escape	12 (3.01%)	3 (2.26%)	0.023	0.880
Complete right bundle branch block	35 (8.77%)	3 (2.26%)	5.441	0.020
Incomplete right bundle branch block	12 (3.01%)	0 (0.00%)	6.188	0.013

**Table 6:** Characteristics of the dynamic electrocardiograms of patients with long R-R intervals (2-3 s vs. >3 s (*n* (%))).

Parameters	Long R-R interval = 2-3 s (*n* = 245)	Long R-R interval >3 s (*n* = 154)	*χ* ^2^	*P*
Second-degree atrioventricular block (*n* = 45)	40 (16.33%)	5 (3.25%)	14.887	0.001
Paroxysmal atrial tachycardia (*n* = 35)	30 (12.24%)	5 (3.25%)	8.476	0.004
Paroxysmal atrial flutter (*n* = 68)	48 (19.59%)	20 (12.99%)	2.469	0.116
Junctional escape beats (*n* = 24)	16 (6.53%)	8 (5.19%)	0.109	0.741
Ventricular escape beats (*n* = 15)	10 (4.08%)	5 (3.25%)	0.068	0.795
Linking phenomenon (*n* = 8)	5 (2.04%)	3 (1.95%)	0.025	0.876
Transient ventricular arrest (*n* = 15)	15 (6.12%)	0 (0.00%)	8.178	0.004
Accelerated ventricular escape (*n* = 12)	8 (3.27%)	4 (2.60%)	0.006	0.937
Complete right bundle branch block (*n* = 35)	35 (14.29%)	0 (0.00%)	22.363	0.001
Incomplete right bundle branch block (*n* = 12)	12 (4.90%)	0 (0.00%)	6.188	0.013

## Data Availability

The data used to support the findings of this study are available from the author upon request.

## Supplementary Materials

Supplementary Materials Supplementary Table 1: frequency of long R-R intervals in variable time periods in patients with nonvalvular atrial fibrillation. The statistical test used: Kruskal–Wallis rank-sum test for independent samples. Supplementary Table 2: frequency of long R-R intervals in variable time periods in patients with nonvalvular atrial fibrillation. The statistical test used: pairwise comparisons using Bonferroni correction. Supplementary Figure 1: at 2:38 am, long RR intervals of 1.5 and 2.0 s appeared after the 4th and 5th atrial fibrillation QRS wave, which was considered as the conducted waves and subsequently recovered. Supplementary Figure 2: at 5:20 am, the heart rate gradually accelerated and a long RR interval of 2.3 s appeared after the 7th atrial fibrillation QRS wave, which was considered as the concealed conduction. The rhythm was reformed and conduction was restored, with no discernible sleep and nonsleep phase discrimination. Supplementary Figure 3: NVAF dynamic electrocardiogram recorded long R-R intervals (asystole) that occurred only during nocturnal sleep periods and not during daytime. Increased vagal tone was considered as the underlying mechanism. Supplementary Figure 4: persistent atrial fibrillation with a 24 h mean heart rate of 53/min, all occurring with long R-R (asystole) and apparent at night. Increased vagal tone and/or concealed or interfered atrioventricular node conduction were considered as the possible underlying mechanism. This observation was also frequent during the daytime, suggesting concealed conduction with interfered and/or combined conduction block in the atrioventricular node. Supplementary Figure 5: at 10:53, a long R-R of 5.7 s was observed after the discontinuation of atrial fibrillation, and the first QRS wave that appeared subsequently was a junctional escape beat. Following that, sinus rhythm recovered with long R-R intervals, suggesting that the “overdrive suppression” in atrial fibrillation renders the sinus node more suppressed or dysfunctional. Supplementary Figure 6: at 10:24, a long R-R of 4.07 s was observed after the discontinuation of atrial fibrillation, with “overdrive suppression” considered as the possible mechanism. The first QRS that appeared subsequently was a sinus rhythm, followed by atrial premature beats with differential conduction and in the form of a complete right bundle branch block waveform. According to the law of bigeminy, atrial premature beats recurred thereafter but did not propagate inferiorly, leading to reoccurrence of the long R-R of 1.53 s and to a concealed conduction, resulting in an abnormal disconnection of the penultimate QRS. Supplementary Figure 7: at 12:45, the termination of atrial fibrillation with one premature ventricular beat after a junctional escape beat resulted in a long RR interval, with atrioventricular junctional extrasystolic action considered as the possible underlying mechanism. The premature ventricular beats produced the results of complete compensatory intermittent and concealed conduction. The QRS wave before restoring to sinus rhythm was a junctional escape, suggesting sinus node suppression and dysfunction. Supplementary Figure 8: at 5:01, the patient reverted to atrial fibrillation that was preceded by a second-degree type I atrioventricular block with a long R-R >2 s of more than three beats, which was not associated with sleep. The patient was diagnosed with atrial fibrillation combined with second-degree atrioventricular block, given the average ventricular rate at onset was less than 40 bpm. Supplementary Figure 9: at 5:01, the patient was in sinus rhythm with second-degree AVB and high AVB (same patient in Supplementary Figure 8). Supplementary Figure 10: at 11:00, slow-type atrial fibrillation with a mean ventricular rate of less than 40 bpm was observed. Atrial fibrillation was associated with long R-R intervals of >2 s for more than 3 beats, independent of sleep. This was considered as atrial fibrillation with second-degree AVB (same patient in Supplementary Figure 8).
